# Clinical Efficacy, Healing Efficacy, and Safety Analysis of Skin Orbicularis Oculi Muscle Combined with Tissue Flap for Eyelid Trauma

**DOI:** 10.1155/2022/3466070

**Published:** 2022-05-20

**Authors:** Jie Chen, Chao Xiao, Na Su, Yubo Han, Zhai Liang, Chao Han, Wenjuan Yu

**Affiliations:** ^1^Medical Cosmetology Department, The Second Affiliated Hospital of Xi'an Medical College, Xi'an 710061, China; ^2^Department of Plastic Surgery, The Second Affiliated Hospital of Zhejiang Chinese Medical University, Hangzhou 310000, China

## Abstract

This study investigates the efficacy, healing efficiency, and safety of skin orbicularis oculi muscle combined with tissue flap repair for eyelid trauma patients. According to the different methods of surgical intervention, this study chooses 78 cases of eyelid injury patients. This study sets up the joint intervention group and the routine repair group, including the joint intervention group adopting the orbicularis oculi muscle skin of composite tissue flap to repair surgery. The routine repair group is treated by conventional repair skin flap transfer operation. Spearman correlation coefficient is used to analyze the correlation between postoperative healing of eyelid trauma patients and quality of life (SF-36) and self-image satisfaction (BIS) scale scores. The surgical intervention of skin orbicularis oculi muscle combined with tissue flap for patients with eyelid trauma has a better plastic repair effect in clinical practice. It can also effectively reduce the risk of postoperative complications, which is conducive to improve the postoperative quality of life and self-image satisfaction of patients.

## 1. Introduction

The eyelids ahead are vulnerable to external damage, and the damaged parts often harmful are bigger. Eyelid part muscle table damage on appearance brings bad influence to the patient, which will be more severe eyelid dysfunction in severe cases. It not only influences the patient's quality of life but also brings psychological shadow to patients [1, 2]. Periocular skin tissue is soft and thin due to its particularity, which is difficult to repair [3, 4]. In the past, conventional flap transfer repair is mostly used for the treatment of patients with eyelid injury. Although it had certain clinical efficacy, patients' satisfaction evaluation of its cosmetic effect is low, indicating that the traditional surgical method still had certain limitations [5]. Orbicularis oculi muscle composite tissue skin flap surgery is the type of repair operation for clinical emerging in recent years, a clinical specialist is used in the treatment of ocular malignant tumor patients, the clinical curative effect is higher, and it is helpful to the eyelid function in patients with lower risk of complications and have rapid recovery in the short term, but there are few operation studies on eyelid injury [6]. Patients with eyelid trauma in our hospital are selected as the research objects in this study, aiming to explore the application effect of skin orbicularis oculi muscle composite tissue flap repair.

A total of 78 cases of eyelid trauma patients admitted to our hospital from January to June 2021 are selected. According to different surgical intervention methods, the combined intervention group and the conventional repair group are established, respectively, with 39 cases in each group. In the combined intervention group, there are 22 males and 17 females, aged from 21 to 56 years old, with an average of (37.26 ± 10.92) years old. The damaged eyelid area ranged from 2.11 to 13.25 cm^2^, with an average of (7.64 ± 3.00) cm^2^. Body mass index (BMI) ranged from 18.75 to 26.82 kg/m^2^ with an average of (23.03 ± 2.45) kg/m^2^. In the conventional repair group, there are 25 males and 14 females, aged 22–54 years, with an average of (34.92 ± 10.23) years; eyelid damaged area ranged from 1.95 to 13.17 cm^2^, with an average of (7.07 ± 3.32) cm^2^, BMI value (19.05–27.06) kg/m^2^, and average (23.47 ± 2.10) kg/m^2^. There are no significant statistical differences in baseline data of patients between the two groups, including gender, age, eyelid damaged area, and BMI (all *P* > 0.05), which confirm that the comparison between groups is scientific and reasonable.

Inclusion criteria are as follows: after admission, all patients are identified as external eyelid avulsion after clinical diagnosis and identification by specialists; the clinical manifestations of the patients are consistent with the clinical operation indications; complete clinicopathological data of patients; and patients with good clinical compliance and high degree of cooperation can cooperate with this study until the end of the study.

Exclusion criteria are as follows: patients with contraindications related to surgery and clinical anesthesia; patients with blood system diseases or signs of coagulopathy; patients with malignant tumor diseases; patients with serious organic dysfunction such as the liver and kidney; and quit the study for various reasons.

The remainder of this study is organized as follows. The related work is described in Section 2.  Section 3 presents the experimental method.  Section 4 provides the experimental result, and Section 5 illustrates data analysis and result discussion. Finally, the conclusions of this study are given in Section 6.

## 2. Related Work

Eyelid injury in patients is mostly caused by external force, which damages part of eyelid muscle surface and surrounding subcutaneous tissue and soft tissue. In serious cases, it will also peel off bone and form open skin avulsion injury. The main characteristics of eyelid injury in clinical practice are more bleeding and irregular edge, so it is difficult to repair [7]. For specialists, in the process of making treatment plans for patients, they should not only pay attention to the effect of plastic repair of patients' damaged areas but also pay attention to the function of patients' eyelids, so as to ensure that patients can get all-round rapid recovery in a short period of time [8].

In the past, conventional blepharoplasty and repair surgery are mostly achieved by arbitrary flap transfer, and the specific step is to select a flap around the patient's eyelid according to the location of eyelid injury and cover the damaged area [9]. However, studies have shown that after traditional conventional surgery, patients do not get a good prognosis and are prone to other complications, such as appearance scar, lack of overall aesthetic feeling, and skin pigmentation, which seriously affect the appearance aesthetics and clinical satisfaction of patients [10]. In addition, eyelid skin defect is also prone to corneal injury, which is mainly because eyelid injury leads to the loss of effective corneal protection, and patients' eyes are at increased risk of external stimulation and bacterial damage. In severe cases, it may lead to exposed keratitis, which seriously threatens patients' visual function [11].

## 3. The Experimental Method

Before surgery, all subjects are photographed at the damaged site. The attending clinical physician formulated a targeted surgical plan according to the lesion range and surrounding normal eye tissue and clarified the location of surgical incision and the lesion resection range. Before the patient entered the operating room, the medical staff communicated with the patient and his/her family about the possible conditions and precautions during the operation and began the operation with the consent of the patient and his/her family. The operating room is routinely disinfected before surgery, and local anesthesia is used after the specific resection range of the patient's eyelid is determined. Patients with corneal epithelial injury are treated with repair before surgery. Patients with lamellar/full-thickness corneal injury and lacrimal canaliculi injury are treated with simultaneous surgical suture. Among them, patients in the conventional repair group are treated with traditional flap transfer repair. According to the eyelid injury of patients, patients with damaged area >2 cm^2^ are treated with A-T rotating composite flap repair and patients with damaged area ≤2 cm^2^ are treated with a-T flap repair. The joint intervention group is treated by composite tissue flap to repair the skin through orbicularis oculi muscle surgery, according to the situation in patients with eyelid injury, patients with orbital damaged area 2 cm^2^ or less on leather fat tissue orbicularis oculi muscle compound preparation and organization of the effective and the angular and patients with nasal root are fixed operation, using 6–0 polyglycolic acid absorption line for patients of damage and meibomian suture. For patients with eyelid damaged area >2 cm^2^, preparation of tissue flap and at the same time, the above mentioned methods to the lateral canthus of excessive movement part of orbicularis oculi muscle to cut short the operation, the 6–0 polyglycolic acid absorption line for patients of damage and meibomian suture, outside until the upper eyelid above, and ensure the normal function of the orbicularis oculi muscle. The excess orbital adipose tissue is then removed along the lower eyelid, and the skin flap of the complex tissue is moved from the inner canthus to the nasal root.

A follow-up survey is conducted 3 months after surgery, and the patients' quality of life is assessed by the SF-36 health survey. The higher the score, the better the quality of life [12]. Self-image scale (BIS) score evaluated 'patients' image self-identity, and the higher the score, the lower the self-image identity [13].

Grade C healing: wound festering infection, wound healing efficiency is low, and healing after treatment. Grade B healing: the wound healed well, and there are no signs of suppuration around the wound, but mild to moderate inflammation. Grade A healing: the wound healing efficiency is high, and no other complications are observed [14].

SPSS 26.0 statistical software is used to analyze and process the data. After the measurement data are verified and confirmed to be in line with normal distribution, they are expressed as mean ± standard deviation $\left(\bar{x}\pm s\right)$ by the *t*-test, count data by (*n*, %) by the *χ*^2^ test, and grade data by ridit analysis and *U* test. Spearman correlation coefficient is used to analyze the correlation between postoperative healing and quality of life (SF-36) and self-image satisfaction (BIS) scale scores of patients with eyelid trauma, and *P* < 0.05 indicates statistically significant differences.

## 4. The Experimental Results

### 4.1. Comparison of the Incidence of Postoperative Complications

The number of cases of eyelid eversion, varus, and edema in the combined intervention group is lower than the conventional repair group, and the total incidence of complications decreased significantly than the conventional repair group (*P* < 0.05).  Table 1 provides the comparison of postoperative complications.

### 4.2. Comparison of the Healing of the Damaged Site 3 Months after Surgery

Three months after surgery, wound healing in the combined intervention group is significantly better than that in the conventional repair group (*P* < 0.05).  Table 2 provides the comparison of healing of the damaged site between the two groups 3 months after surgery.

### 4.3. Comparison of SF-36 and BIS Scores before and after Surgery

Before surgery, there are no significant differences in SF-36 and BIS scores between the two groups (*P* > 0.05). After surgery, the SF-36 score of the two groups increased significantly before surgery, and the combined intervention group increased significantly than that of the conventional repair group (*P* < 0.05). After surgery, the BIS score of the two groups decreased significantly than that before surgery, and the score of the combined intervention group decreased significantly than the conventional repair group (*P* < 0.05).  Table 3 provides the comparison of SF-36 and BIS scores.

### 4.4. Analysis of the Correlation between Healing Degree and SF-36 and BIS Score

Spearman correlation coefficient analysis shows that the degree of postoperative healing of patients with eyelid injury is positively correlated with SF-36 score, and the degree of postoperative healing of patients with eyelid injury is negatively correlated with BIS score (*P* < 0.05).  Table 4 provides the correlation of healing degree with SF-36 and BIS scores.

## 5. The Experimental Result Discussion

The results show that the intervention of the orbicularis oculi muscle combined with tissue flap to repair skin operation is applied to the eyelid injury and surgical treatment of patients and can effectively reduce the risk of postoperative adverse complications, postoperative wound healing of 3 months more for routine repair surgery patients, postoperative patients life quality, and self-image satisfaction that has improved significantly. It is confirmed that skin orbicularis oculi muscle combined with tissue flap repair has higher clinical efficacy and safety and higher healing efficiency. The reason for the above results may be that traditional repair methods often only focus on anatomical reduction and fail to focus on details. Overall eyelid repair, including repair of orbicularis oculi muscle and periocular skin, is crucial to the appearance and function of the eyelid. Joint intervention before operation will meibomian skin orbicularis oculi muscle as a whole; the orbicularis oculi muscle skin complex, in operation, at maximum limit guaranteed the cut edge of the skin and orbicularis oculi muscle fit closely, in guarantee close their eyes when no concave traces; dynamic heavy eyelid folds at the same time guarantee the orbicularis oculi muscle support for meibomian former skin tissue nutrition, rapid postoperative recovery. Edema is not obvious. In the treatment of the upper edge of the incision, the orbicularis oculi muscle is always retained slightly more than the skin edge of the upper lip of the incision, so that the orbicularis oculi muscle at the upper and lower edges can grow in alignment after suturing, ensuring the continuity of the orbicularis oculi muscle. In other words, the beautiful double eyelid shape is formed, the continuous physiological structure of orbicularis oculi muscle is restored, postoperative recovery is accelerated, and the metabolism of premeibomian tissue is beneficial. In addition, this study aims at patients healed and launches the correlation degree and life quality and self-image satisfaction research. It is found that patients with wound healing and their satisfaction with the quality of life and self-image are closely related. It also fully confirms the effective intervention operation and helps to increase the efficiency of the patients and improve the prognosis of patients at the same time.

## 6. Conclusion

In conclusion, the application of skin orbicularis oculi muscle composite tissue flap for eyelid avulsion has a significant effect, which can effectively reduce complications and improve aesthetic satisfaction. However, there are still areas to be improved in this study. First, eyelid injury is rarely seen in clinical practice, so the sample size selected in this study is very limited, and the follow-up investigation of patients in this study only lasts for three months, so the follow-up time of patients' prognosis after surgery should be extended.

## Figures and Tables

**Table 1:** Comparison of postoperative complications (*n*, %).

Group	Eyelid ectropion	Eyelid varus	Occurrence edema	Total occurrence ratio
Combined intervention group (*n* = 39)	1 (2.56)	2 (5.13)	0 (0.00)	3 (7.69)
Routine repair group (*n* = 39)	5 (12.82)	4 (10.26)	2 (5.13)	12 (30.77)
*X* ^2^	—	—	—	6.686
*P*	—	—	—	0.010

**Table 2:** Comparison of healing of the damaged site between the two groups 3 months after surgery (*n*, %).

Group	Class A healing	Class B healing	Class C healing
Combined intervention group (*n* = 39)	34 (87.18)	3 (7.69)	2 (5.13)
Routine repair group (*n* = 39)	19 (48.72)	10 (25.64)	10 (25.64)
*U*	4.769		
*P*	＜0.001		

**Table 3:** Comparison of SF-36 and BIS scores $\left(\bar{x}\pm s\right)$.

Group	SF-36 scale		The BIS score	
	Before the operation	After the operation	Before the operation	After the operation
Combined intervention group (*n* = 39)	62.41 ± 2.41	77.21 ± 4.58^*∗*^	15.10 ± 1.16	7.52 ± 0.66^*∗*^
Routine repair group (*n* = 39)	61.81 ± 1.78	69.80 ± 3.04^*∗*^	15.23 ± 1.04	9.20 ± 0.86^*∗*^
*t*	1.251	8.418	−0.521	−9.678
*P*	0.215	＜0.001	0.604	＜0.001

**Table 4:** Correlation of healing degree with SF-36 and BIS scores.

	Degree of patient healing	
	*rs*	*P*
SF-36 scale	0.704	<0.001
The BIS score	−0.810	<0.001

## Data Availability

The data used to support the findings of this study are available from the corresponding author upon request.
